The article "Protective Effects of Shen-Yuan-Dan Capsule against Ischemia/Reperfusion Injury in Cardiomyocytes by Alleviating Endoplasmic Reticulum Stress" was published in 2022. Journal: Evid Based Complement Alternat Med.

# Protective Effects of Shen-Yuan-Dan Capsule against Ischemia/Reperfusion Injury in Cardiomyocytes by Alleviating Endoplasmic Reticulum Stress

**DOI:** 10.1155/2022/7775876

**Published:** 2022-07-06

**Authors:** Tong Tong, Zhihai Yang, Jiaxing Chen, Tao Gong, Hongxu Liu

**Affiliations:** ^1^Department of Cardiology, Beijing Hospital of Traditional Chinese Medicine, Capital Medical University, Beijing 100010, China; ^2^Beijing Institute of Traditional Chinese Medicine, Beijing 100035, China

## Abstract

**Objective:**

Endoplasmic reticulum (ER) stress leads to the accumulation of misfolded proteins and an active unfolded protein response (UPR). If the ER stress is not resolved, the UPR triggers activation of the apoptotic cell death program. It has been shown that ischemia/reperfusion (I/R) injury can induce apoptosis via the ER stress pathway. We previously found that Shen-Yuan-Dan capsule (SYDC), a widely used traditional Chinese medicine, reduces I/R injury. Here, we investigated whether SYDC protects against cardiomyocyte apoptosis by reducing ER stress during I/R injury and. if so, explored its mechanism of action.

**Methods:**

We use forty male Wistar rats to prepare the SYDC pharmacological serum. An I/R injury model was established using cultures of neonatal rat ventricular myocytes where cells were exposed to 2 h of reduced oxygenation followed by 4 h of normal oxygenation. After treatment of cultured cells with serum containing SYDC for 4 h, reverse transcription polymerase chain reaction and western blotting were performed to assess the expression levels of target molecules.

**Results:**

Ischemia/reperfusion (I/R) clearly decreased cell viability. Treatment of cells with SYDC in serum (5% and 10%) increased cell viability compared with control serum-treated I/R cardiomyocytes. The mRNA levels of glucose-regulated protein 78 (Grp78), C/EBP homologous protein (CHOP), and caspase-12 were significantly upregulated in the I/R group. The mRNA levels of Grp78, CHOP, and caspase-12 were significantly decreased in the 5% and 10% SYDC groups compared to the I/R group. The protein expression levels of Grp78, CHOP, and caspase-12 were significantly upregulated in the I/R group. Treatment of I/R cardiomyocytes with 5% or 10% SYDC reduced the expression levels of CHOP and caspase-12, while the control serum did not show this effect.

**Conclusions:**

These findings demonstrate that SYDC alleviates ER stress and prevents ER stress-induced apoptosis via the CHOP-dependent pathway.

## 1. Introduction

The endoplasmic reticulum (ER) is an important organelle in eukaryotic cells that regulates protein synthesis, protein folding and trafficking, cellular responses to stress, and intracellular calcium (Ca^2+^) levels [1, 2]. Triggers for ER stress (ERS) include nutritional deficiency, abnormal protein transport, and dysregulated disulfide bond formation [3]. If ERS persists, cellular apoptosis occurs.

The article "Protective Effects of Shen-Yuan-Dan Capsule against Ischemia/Reperfusion Injury in Cardiomyocytes by Alleviating Endoplasmic Reticulum Stress" was published in 2022. Journal: Evid Based Complement Alternat Med.

Shen-Yuan-Dan capsule (SYDC) is a widely used traditional Chinese medicine. Data from previous studies suggest that oral supplementation with SYDC for 4 weeks not only relieves the symptoms of patients with angina but also promotes the recovery of cardiac dysfunction in these patients [4, 5]. We also demonstrated that SYDC reduces myocardial infarct size [6], promotes endothelial function [7], inhibits oxidative injury [8], and protects against myocardial ischemia/reperfusion (I/R) injury in both *in vivo* and *in vitro* models via activation of the phosphatidylinositol 3-kinase/Akt (PI3K/Akt) pathway [9]. However, the underlying mechanisms by which SYDC reduces myocardial cell apoptosis remain unclear. We hypothesized that SYDC may inhibit apoptosis in cardiomyocytes by alleviating ER stress. Therefore, in the present study, we determined the effects of SYDC on the expression of glucose-regulated protein 78 (Grp 78) and the apoptosis factors C/EBP homologous protein (CHOP) and caspase-12 to investigate the possible mechanisms by which SYDC protects myocyte apoptosis by alleviating ER stress during I/R injury.

## 2. Materials and Methods

### 2.1. Animals and Chemicals

Forty male Wistar rats weighing 200–220 g were used to prepare the SYDC pharmacological serum. Rats were divided into two groups, namely, an SYDC and a saline control. Neonatal (1- to 3-day-old) Wistar rats were used as a source of neonatal cardiomyocytes for cell culture experiments. All animals were purchased from Charles River Laboratories (Beijing, China). All experimental procedures were performed in accordance with the guidelines of the Animal Care and Use Committee, Beijing TCM Hospital, Capital Medical University (Beijing, China). All experiments conformed to the National Institutes of Health Guide for the Care and Use of Laboratory Animals.

Cell counting kit-8 (CCK-8) was purchased from Dojindo Laboratories (Kumamoto, Japan). Trizol, phosphate-buffered saline (PBS), 5-bromo-2′-deoxyuridine (Brd-U), trypsin, and collagenase were purchased from Sigma Aldrich (St. Louis, MO, USA). Fetal bovine serum and Dulbecco's modified Eagle's medium (DMEM)-F12 were purchased from Hyclone (Logan, UT, USA), and TransScript® One-Step gDNA Removal and cDNA Synthesis SuperMix and TransStart® Top Green qPCR SuperMix were purchased from TransGen Biotech (Beijing, China). Penicillin-streptomycin mixture was obtained from the Chinese Academy of Medical Sciences and Peking Union Medical College Institute of Biomedical Engineering (Beijing, China).

The article "Protective Effects of Shen-Yuan-Dan Capsule against Ischemia/Reperfusion Injury in Cardiomyocytes by Alleviating Endoplasmic Reticulum Stress" was published in 2022. Journal: Evid Based Complement Alternat Med.

### 2.2. Preparation of SYDC Pharmacological Serum

SYDC pharmacological serum was obtained as previously described [9]. In brief, 50 Wistar rats weighing 200–220 g were divided into two groups, namely, an SYDC and a saline control. SYDC (10 mL/kg) or saline (10 mL/kg) were administered by oral gavage twice a day for 5 days. One hour after the final oral gavage, blood was drawn from the abdominal aortic artery from each animal and then centrifuged at 3000 rpm for 10 min. The sera collected from animals in each group were combined, inactivated at 56°C for 30 min, transferred to 4 mL tubes, and stored at −80°C. Before all experiments, both SYDC and control sera were diluted to 5% and 10% (v/v) with DMEM/F12 culture medium.

### 2.3. Culture of Neonatal Cardiomyocytes

Neonatal cardiomyocytes from 1–3-day-old Wistar rats were cultured as described previously [10]. In brief, cardiomyocytes were isolated from newborn rats using the trypsin and collagenase method and differential attachment and Bru-U to minimize fibroblast contamination. After 48 h of culture in DMEM/F12 containing 10% FBS and 1% penicillin-streptomycin at 37°C and 5% CO_2_, cardiomyocytes were transferred to serum-free DMEM/F12. Cells were randomly and homogeneously distributed into six groups, as follows. Control group: cardiomyocytes were incubated for 24 h at 37°C, containing 95% air and 5% CO_2_. I/R group: after replacing the medium with glucose-free Earle's balanced salt solution, the cells were cultured in a trigas incubator (95% N_2_ + 5% CO_2_) for 2 h (ischemia). Thereafter, Earle's solution was replaced with DMEM/F12 containing 10% FBS, and the cells were moved into an incubator (95% air + 5% CO_2_) for 4 h (reperfusion) to establish the I/R injury model. In the other four groups, after the ischemia phase, Earle's balanced salt solution was replaced with DMEM/12 supplemented with 5% or 10% SYDC pharmacological serum (5% SYDC, 10% SYDC) or DMEM/12 supplemented with 5% or 10% control serum (5% control and 10% control).

### 2.4. Cell Counting Kit (CCK8) Assay

Myocardial cells were cultured in a 96-well plate at a density of 2 × 10^5^ cells/well. At the end of the reoxygenation period, the CCK8 assay was performed according to the manufacturer's instructions; absorbance was measured at 450 nm.

### 2.5. Real-Time Quantitative Polymerase Chain Reaction (qPCR)

RNA was isolated from cardiomyocytes using Trizol reagent and cDNA prepared using TransScript® One-Step gDNA Removal and cDNA Synthesis SuperMix and TransStart® Top Green qPCR SuperMix, according to the manufacturer's instructions. The primer sequences used for PCR are listed in Table 1. The thermal cycle reaction was executed as follows: 95°C for 3 min, followed by 40 cycles at 95°C for 30 s and 60°C for 30 s. The levels of each target were determined from the relative standard curves.

The article "Protective Effects of Shen-Yuan-Dan Capsule against Ischemia/Reperfusion Injury in Cardiomyocytes by Alleviating Endoplasmic Reticulum Stress" was published in 2022. Journal: Evid Based Complement Alternat Med.

### 2.6. Western Blotting

The cardiomyocytes were rinsed, harvested in ice-cold PBS, and pelleted by centrifugation. Following this, the cardiomyocytes were washed and resuspended in extraction buffer (RIPA : PMSF : cocktail : phosphatase inhibitors = 100 : 1 : 1 : 1), maintained at a constant agitation for 30 min at 4°C, after which the lysate was centrifuged at 12,000 × *g* for 30 min in a 4°C precooled centrifuge. The supernatant was gently transferred to a fresh tube kept on ice, and the pellet was discarded.

The supernatant was mixed with 5x loading buffer and heated for 15 min at 95°C. Proteins (100 *μ*g) were loaded into the wells of SDS-PAGE gel. After electrophoresis, proteins were electrophoretically transferred to a PVDF membrane and then blocked with 3% bovine serum albumin for 2 h. The blots were then incubated with antibodies against Grp78 (1 : 1000), caspase-12 (1 : 1000), and CHOP (1 : 1000) in TBST. The membrane was washed three times with TBST for 10 min each time and then rinsed with TBS. Membranes were incubated with the appropriate secondary antibody at room temperature for 2 h. Immunoreactive protein bands were detected using the ECL detection kit (Applygen Technologies Inc.). Images were quantified by scanning the films, and band densities were determined using ImagePro software.

### 2.7. Statistical Analysis

All data are expressed as the mean ± standard error of the mean (SEM). Differences between groups were analyzed using a one-way analysis of variance (ANOVA) with a Student–Newman–Keuls post hoc test. For all analyses, *P* < 0.05 was considered statistically significant. All statistical analyses were performed using SPSS software (version 11.0, SPSS Inc., Chicago, IL, USA).

## 3. Results

### 3.1. Effects of SYDC Pharmacological Serum on the Viability of I/R Cardiomyocytes

For the effect of SYDC pharmacological serum on the viability of I/R cardiomyocytes, cardiomyocytes were assessed using a CCK8 assay. The viability of I/R cardiomyocytes in the 5% SYDC pharmacological serum group was significantly higher than that of cells in the other I/R groups (*P* < 0.01) (Figure 1).

### 3.2. Effects of SYDC Pharmacological Serum on ER Stress-Associated Genes

The mRNA levels of ER stress-associated genes (Grp 78, CHOP, and caspase-12) were measured by real-time qPCR. The results showed that the mRNA levels of Grp 78, CHOP, and caspase-12 were significantly upregulated in the I/R group compared to the control group (*P* < 0.01). The mRNA levels of Grp 78, CHOP, and caspase-12 were significantly decreased in the 5% SYDC group and the 10% SYDC group (*P* < 0.05 and *P* < 0.01, respectively). Compared to the 10% control serum-treated group, the levels of Grp78 and caspase-12 were markedly decreased in the 10% SYDC group (*P* < 0.05). The levels of CHOP in the 5% SYDC group were significantly lower than in the 5% control serum-treated group and the 10% SYDC group (*P* < 0.01) (Figure 2).

The article "Protective Effects of Shen-Yuan-Dan Capsule against Ischemia/Reperfusion Injury in Cardiomyocytes by Alleviating Endoplasmic Reticulum Stress" was published in 2022. Journal: Evid Based Complement Alternat Med.

### 3.3. Effect of SYDC Pharmacological Serum on the Expression Levels of ER Stress-Associated Proteins in I/R Cardiomyocytes

Western blot was used to assess the expression of ER chaperone proteins in I/R cardiomyocytes. The results showed that expression levels of Grp78, CHOP, and caspase-12 were significantly upregulated in the I/R group compared to the control group (*P* < 0.05 or *P* < 0.01). Treatment of I/R cardiomyocytes with 5% or 10% SYDC for 2 h induced a downregulation of Grp78, CHOP, and caspase-12, while the control serum did not show this effect (*P* < 0.05 or *P* < 0.01). There was no significant difference between the 5% and 10% SYDC groups (Figure 3).

## 4. Discussion

Traditional Chinese medicine is widely used to treat many kinds of cardiovascular and metabolic diseases. Previously, we showed that SYDC, a traditional Chinese medicine prescription, has beneficial effects in protecting the ischemic myocardium from I/R injury and inhibiting apoptosis in I/R cardiomyocytes [9]. It consists of eight crude Chinese medicinal agents named *Salvia miltiorrhiza* Bge, *Astragalus membranaceus* Bge, root of *Pilose Asiabell, Radix Scrophulariae, Hirudo nipponica* (Whitman)*, Lumbricus, Eupolyphagasinensis* (Walker), and *Rhizoma Corydalis.*

The myocardial cell is extremely sensitive to oxygen deficit, which makes it vulnerable injury from hypoxia. In our previous studies [9], after 2 h of hypoxia and 4 h of hypoxia, the cell serum activities of LDH and CK-MB were significantly increased in H/R group as compared with the sham group, and the viability of H/R group cells was decreased compared with the normal group. The study has suggested that myocardial cells undergo I/R injury after modeling.

The ER is an organelle that is sensitive to a variety of different stimulants. Stimulating factors such as ischemia, anoxia, nutrient deficiency, tunicamycin, Ca^2+^-ATPase inhibitors, and viral infections can cause an increase in protein synthesis. ER stress is associated with the accumulation of unfolded or misfolded proteins. In response to ER stress conditions, a self-protective mechanism called the unfolded protein response (UPR) is activated. Over the last decade, it has become clear that UPR is activated in response to hypoxia [11] and may play an important role in I/R injury [12–14] and is related to cellular apoptosis [15]. Research has suggested that myocardial I/R injury leads to massive death of cardiomyocytes and plays an important role in the development of coronary heart diseases (CHDs) [16, 17]. While I/R clearly decreased cardiomyocyte viability, culturing I/R cells in the presence of SYDC pharmacological serum (5% and 10%) resulted in a maintenance of cell viability at a high level. While cardiomyocytes exposed to control sera (5% and 10%) also exhibited improved viability compared with the I/R group, the protective effect of serum alone was not as beneficial as that of SYDC pharmacological serum.

The article "Protective Effects of Shen-Yuan-Dan Capsule against Ischemia/Reperfusion Injury in Cardiomyocytes by Alleviating Endoplasmic Reticulum Stress" was published in 2022. Journal: Evid Based Complement Alternat Med.

The UPR results in the inhibition of proteins synthesis and the increased expression of molecular chaperones in order to alleviate overload of the ER and maintain cell survival [12]. It is believed that most of the initial UPR responses aim to adapt to ER stress and help the ER to restore homeostasis [18]. While moderate ER stress plays a positive role in maintaining ER function and homeostasis by enhancing the protein folding capacity, with the increased expression of the ER chaperones Grp78 and Grp94, excessive ER stress can cause cell injury, death, and apoptosis [19]. Grp 78, an indicator of ER stress, is markedly upregulated during ER stress. Prolonged ERS leads to the initiation of apoptotic processes mediated by CHOP and caspase-12 [20]. In our study, the levels of Grp 78 were significantly upregulated, suggesting that I/R injury can trigger cell apoptosis via the ER stress pathway. After intervention with pharmacological serum of SYDC at different concentrations (5% and 10%), but not control serum, the levels of Grp78 were significantly downregulated as assessed by both RT-PCR and western blotting.

During the UPR, Grp 78 combines with unfolded or misfolded proteins and helps them fold correctly. Overexpression of Grp78 is induced when there is an excess of misfolded and unfolded proteins in the ER, activating the expression of PERK1, IRE1, and ATF6 [11]. Upregulation of CHOP, phosphorylation of IRE1, and activation of Janus N-terminal kinase (JNK) lead to cell apoptosis in the end phase [13]. Caspase-12 is located on the ER membrane and is activated only by ER stress [21, 22].

We found that by both RT-PCR and western blot analysis, compared with the control group, the gene and protein expression levels of CHOP and caspase-12 in the I/R group increased significantly. After intervention with SYDC serum, the levels of CHOP and caspase-12 were significantly reduced. This result is consistent with our previous experiments on the activity of cardiomyocytes.

The article "Protective Effects of Shen-Yuan-Dan Capsule against Ischemia/Reperfusion Injury in Cardiomyocytes by Alleviating Endoplasmic Reticulum Stress" was published in 2022. Journal: Evid Based Complement Alternat Med.

In conclusion, the results of the present study demonstrate that SYDC is effective in its downregulating endoplasmic reticulum-related factors and protecting cardiomyocytes from I/R-induced apoptosis. This study suggests that SYDC may reduce myocardial injury and complications in patients with coronary heart disease, and so this kind of treatment may bring huge benefits for patients with coronary heart disease. There are still some shortcomings in this study. There was no clear dose-effect relationship of SYDC, which may be related to the small sample size of the experimental group.

## Figures and Tables

**Figure 1:** Effects of SYDC pharmacological serum on the viability of I/R cardiomyocytes. ^*∗∗*^*P* < 0.01, compared with the I/R group; ^△△^*P* < 0.01, compared with the 5% control group; ^##^*P* < 0.01, compared with the 10% control group.

**Figure 2:** Effects of SYDC pharmacological serum on the levels of ER stress-associated genes. (a) The mRNA levels of glucose-regulated protein 78 (Grp 78) in cardiomyocytes. (b) The mRNA levels of C/EBP homologous protein (CHOP) in cardiomyocytes. (c) The mRNA levels of caspase-12 in cardiomyocytes. ^*∗*^*P* < 0.05, compared with the I/R group; ^*∗∗*^*P* < 0.01, compared with the I/R group; ^△△^*P* < 0.01, compared with the 5% control group; ^#^*P* < 0.05, compared with the 10% control group; ^▲▲^*P* < 0.01, compared with the 5% SYDC group.

**Figure 3:** Western blot showing the expression levels of Grp78, CHOP, and caspase-12 in cardiomyocytes. Expression of Grp78, CHOP, and caspase-12 in cardiomyocytes. *β*-Actin was used as a loading control. ^*∗*^*P* < 0.05, compared with the I/R group; ^*∗∗*^*P* < 0.01, compared with the I/R group; ^△△^*P* < 0.01, compared with the 5% control group; ^#^*P* < 0.05, compared with the 10% control group; ^##^*P* < 0.01, compared with the 10% control group.

**Table 1:** Primer sequences used in the polymerase chain reaction (PCR).

Gene name	Primer name	Primer	Size
Grp 78	Grp78_Primer_F	CTGGACTGAATGTCATGAGG	66
	Grp78_Primer_R	TATCCAGGCCATATGCAATAG	
CHOP	CHOP_Primer_F	TCCCAAAGCCCTCGCTCTCCA	111
	CHOP_Primer_R	GCTGCGCACTGACCACTCTGTT	
Caspase-12	Casp12_Primer_F	TGGAAGGTAGGCAAGAGTGGC	147
	Casp12_Primer_R	GGTGGGCATCTGGGTCAGTT	
GAPDH	JNK_Primer_F	TGCACCACCAACTGCTTAGC	87
	JNK_Primer_R	GGCATGGACTGTGGTCATGAG	

CHOP, C/EBP homologous protein; GAPDH, glyceraldehyde-3-phosphate dehydrogenase; Grp78, glucose-regulated protein 78.

## Data Availability

The data that support the findings of this study are available from the corresponding author upon reasonable request.
